The article "3D Digital Model of Folk Dance Based on Few-Shot Learning and Gesture Recognition" was published in 2022. Journal: Comput Intell Neurosci.

# 3D Digital Model of Folk Dance Based on Few-Shot Learning and Gesture Recognition

**DOI:** 10.1155/2022/3682261

**Published:** 2022-06-30

**Authors:** Ning Zhang

**Affiliations:** Shandong University of Arts, Jinan 250000, China

## Abstract

Folk dance is a very unique local culture in China, and dances in different regions have different characteristics. With the development of 3D digital technology and human gesture recognition technology, how to apply it in folk dance is a question worth thinking about. So, this paper recognizes and collects dance movements through human body detection and tracking technology in human gesture recognition technology. Then, this paper writes the data into the AAM model for 3D digital modeling and retains the information by integrating the manifold ordering. Finally, this paper designs a folk dance learning method combined with the Few-Shot learning method. This paper also designs a data set test experiment, an algorithm data set comparison experiment, and a target matching algorithm comparison experiment to optimize the learning method designed in this paper. The final results show that the Few-Shot learning method based on gesture recognition 3D digital modeling of folk dances designed in this paper reduces the learning time by 17% compared with the traditional folk dance learning methods. And the Few-Shot learning method designed in this paper improves the dance action score by 14% compared with the traditional learning method.

## 1. Introduction

Dance is an art with soul. It not only brings beautiful enjoyment to people, but also inherits rich and profound cultural connotations and is a cultural carrier. China is a multiethnic country, ethnic dance is prosperous, and the art of each ethnic group has a long history of development, and all have distinctive dance art culture. Ethnic folk dance is an important artistic carrier in the long history of China since ancient times, and it inherits and develops the cultural origin and artistic orientation of various ethnic groups.

The research on human action cognition, from simple to complex, can be summarized into three levels: mobile vision, action vision, and action vision according to the content of the action. At present, there are two main problems in studying the action vision of video people. One is that, during the recognition process, most of the action frame information in the video will be repeated, or the correlation with action recognition will be very low, the calculation will become complicated, and it will also affect the action. Second, in the process of feature selection and understanding, the main methods include fusing representational and pose-based features. However, the costumes of the stage background and dance moves can be changed, so in many cases, the motion information of the human body cannot be accurately and completely represented in the fusion of the expression information, and the static state of the human body is ignored according to the characteristics of the posture. The Few-Shot learning method based on gesture recognition 3D digital modeling of ethnic dance designed in this paper has great significance for students majoring in ethnic dance, which can allow students to learn ethnic dance very effectively.

The innovation of this paper is as follows: through the method of human body detection and tracking technology in the human body gesture recognition technology, this paper recognizes and collects the movements and human body postures of folk dances. Then, the AAM model is used for 3D digital modeling. In this paper, the information of manifold ordering is integrated and retained. Then, through the analysis, this paper designs a folk dance Few-Shot learning method. In order to optimize the Few-Shot learning method of 3D digital modeling of folk dance based on gesture recognition, this paper also designs a data set test experiment, an algorithm data set comparison experiment, and a target matching algorithm comparison experiment.

## 2. Related Work

Cell line screening has created extensive datasets for learning predictive markers of drug response, but these models are not easily translated to the clinic due to their diverse backgrounds and limited data. Ma J applies a recently developed technique, few-shot machine learning, to train a general neural network model in cell lines that can be adapted to new environments using few additional samples. His main research is based on medical aspects although it combines small sample methods, but it has little relevance in gesture recognition technology. Spectral prediction using deep learning [1, 2] has attracted a lot of attention in recent years. While existing deep learning methods have shown significant improvements in prediction accuracy, there is still considerable room for improvement, currently limited by differences in debris types or instrument settings. Lu Z presented an algorithmic framework to process acceleration and surface electromyography (SEMG) signals for gesture recognition. It includes a novel segmentation scheme, a score-based sensor fusion scheme, and two new features. The framework uses a Bayesian linear classifier and an improved dynamic time warping algorithm [3]. Human gesture recognition plays an important role in many human interaction applications, such as cell phones, health monitoring systems, and human-assisted robots. Electromyography (EMG) is one of the most common and intuitive methods for detecting gestures based on muscle activity. However, EMGs are often overly sensitive to environmental disturbances such as electrical noise, electromagnetic signals, and humidity. Jung P G proposed a new method for muscle activity recognition based on air pressure sensor and air bag. It detects muscle activity by measuring changes in air pressure in air sacs that contact the muscle of interest [4]. Numerous folk dance videos are uploaded online or added to Bollywood movies as situational songs. Classification of folk dance videos is critical for dance education, preservation of cultural heritage, and better customer-oriented service by music companies. Bhatt M proposed a folk dance classification framework. The framework extracts the audio signal from the video, extracts a 125-second segment from the beginning, and further divides it into a set of small segments. It computes Mel-Frequency Cepstral Coefficients (MFCC) and Linear Predictive Coding (LPC) coefficients to generate high-dimensional feature vectors. He uses Principal Component Analysis (PCA) to reduce dimensionality and uses a scale conjugate gradient neural network to classify segments [5]. Maintaining the quality of 3D data in the potentially long chain from digital scan to 3D model deployment is critical for the increasing number of advanced geometric design processes in the mesh domain, including digital fabrication. Centin M proposes an extremely general solution. It handles all previously described problems in a user-friendly way. And it is based on the original multiforward propulsion triangulation technique guided by implicit surfaces and based on the priority mechanism, which greatly reduces the frontal interference [6]. The three-dimensional (3D) revolution promises to transform archaeological practice. Among the techniques that aid in the proliferation of 3D data, photogrammetry facilitates fast and inexpensive digitization of complex subjects in field and laboratory settings. Magnani M discusses how the technique adapts and extends existing document and data visualization routines, while evaluating the opportunities it offers to solve archaeological problems and problems in innovative ways [7]. To sum up, most of the literature is about Few-Shot learning and pose recognition. Although it involves folk dance, the focus is not on the creation of its 3D digital model. So, the next focus of this paper is to combine Few-Shot learning and gesture recognition to perform 3D digital modeling of traditional folk dance.

## 3. Few-Shot Learning Method for 3D Digital Modeling of Folk Dance Based on Gesture Recognition Technology

### 3.1. Human Pose Recognition

#### 3.1.1. Principle of Depth Map Acquisition

Since the release of Kinect [8, 9], depth cameras have received more and more attention. Depth cameras currently in the market can be divided into the following three categories according to technology: structured light-based cameras (SL), time-of-flight cameras (ToF), and stereo vision-based cameras (Stereovision).

#### 3.1.2. Structured Light

The depth acquisition method based on structured light [10] is an active stereo vision technique. A series of known patterns are projected onto the object in turn and deformed according to the object's geometry, viewing the object from different directions. Depth information is extracted by analyzing the distortion of the observed patterns (e.g., differences from original mode), as detailed in Figure 1.

#### 3.1.3. Flight Time

The acquisition method based on the time of flight [11] is to continuously send light pulses of different phases to the object and then use the sensor to receive the light reflected by the object to calculate the round-trip time (i.e., phase difference). A pulse of light is used to obtain the distance between the device and the object. As shown in Figure 2, the red line represents the infrared light wave transmitted to the object, and the infrared component reflected by the sensor is detected.

### 3.2. Human Detection and Tracking Technology

From photo and video streams, human detection techniques [12] extract people. Traditional detection technology [13, 14] and statistical principle detection technology are commonly used in human body detection technology. Human detection techniques based on statistics can be divided into two stages: training and detection. Multiple detected and noise samples are collected during the training phase, positive and negative feature vectors are created, and features are created based on training and classification. The video frames to be detected are scanned one by one in the detection phase. At the corresponding position, a feature is formed, and then the person's target is determined.

So far, the human body detection technology needs to realize the detection of moving objects first, and the optical flow method and the adjacent frame difference method are general. Humans and non-humans are then classified based on the foreground, that is, the ratios and shapes of parts of the human body, or by analyzing the color of human skin against the characteristics of the image. This traditional detection method is not effective for the interference of complex external environment and external objects and is also easily affected by the noise of the underlying image features.

### 3.3. Moving Human Target Detection

Detecting moving objects is viewed as a spatial domain partition of video objects. Specifically, this refers to the detection and separation of regions of people moving independently in the video sequence for each frame. The most common ways of distinguishing are as follows.

Frame Difference Method [15]: the frame difference method is one of the commonly used moving object detection and segmentation methods. The basic idea is to use strong correlations between adjacent frames of an animation sequence in order to detect changes. The algorithm is characterized by high speed and high real-time performance, and changes in light have little effect on the algorithm. However, the segmentation accuracy of moving objects is not guaranteed, and large holes can be simply generated.

Background difference method [16]: the background difference method uses the difference between the current image and the background image to detect moving regions. This method is typically used for background static or slowly changing and provides the most complete characteristic data. However, due to the sensitivity to the interference of irrelevant objects in the scene, many scholars have focused on the research of background update algorithms.

Optical flow method [17]: the optical flow method is an approximate estimation of the plane projection of the two-dimensional image of the three-dimensional motion of the actual sports field scene, lens, target, etc. Its characteristic is that it can deal with the motion of the background more appropriately, but it is sensitive to noise and the calculation is very complicated.

### 3.4. Action Sequence Segmentation

The initial action recognition was only to recognize human movement through the computer, and later, it developed into simple actions including some simple actions, such as walking, running, and jumping. Each video frame sequence contains multiple types of actions, and each type of action contains multiple simple actions. Each simple movement consists of multiple human poses. The consistency and smoothness of various actions are due to the convergence of transition actions. In the case of dance moves, a complete dance performance includes multiple movement groups. Each action group consists of multiple simple actions, such as clips and steps, and simple actions consist of multiple basic poses such as raising hands and kicking feet. Therefore, the purpose of video frame sequence segmentation is to segment human action sequences into small actions. This will keep action sequences as short as possible but contain enough action information to identify the type of action. It is difficult to precisely find the dividing point if the human action is continuous and smooth. This is the main reason why the segmentation of video action sequences is not ideal, and only by extracting key frames for action sequence segmentation cannot achieve the shortest possible data to contain the most human action information. In fact, in most cases of video action recognition research work, we choose to manually process video, such as using manual segmentation to obtain the action sequence of the main data, or planning the action to be collected when collecting data. A whole video is divided into multiple small videos according to simple actions and recorded separately, and then the action sequences formed by all video frames are used for video action recognition].

### 3.5. 3D Digital Modeling

#### 3.5.1. Motion Capture

People look forward to capturing human movements in the most intuitive and natural way. That is, the human body can move freely, and the camera can capture and record motion information just like the human eye. This is what the motion capture system based on computer vision system pursues, and its typical processing process is shown in Figure 3.

#### 3.5.2. Overview of the AAM Model

Active appearance model is a feature point localization method widely used in pattern recognition and computer vision. In the process of establishing the AAM model, the global shape and texture information are fully considered, and the final AAM model can be obtained by modeling the shape and texture respectively, and by instantiating the model. In the process of image matching, the reverse composite method is adopted, which has achieved very good results in real-time and accuracy.

The establishment of AAM model is mainly divided into shape modeling, texture modeling, and the appearance model generated by combining these two models. The instantiation of the model is to map the appearance model to the corresponding shape instance through affine transformation.

The shape model of AAM refers to the ASM model. ASM is a model based on point distribution. It only trains the shape model and lacks the texture model, so the location of the feature points of the face is not accurate. The AAM model can solve this problem very well.

The general modeling object of the AAM model is a nonrigid object, such as a human face, and the main purpose is to describe the object through model parameters (feature points). Then, it can use this description to complete other tasks, such as image alignment, target location, tracking [18, 19], and recognition [20].

Because the active shape model ASM model only counts the shape model, we need to build a texture model that uses the grayscale information of the face to model, which is actually the grayscale value of the pixel. The number of pixels in the shape needs to be transformed to be consistent, and the method used is piecewise linear affine transformation. As shown in Figure 4, it is a piecewise linear affine transformation.

The calculation method of piecewise linear affine transformation [21] is shown in Figure 5:

#### 3.5.3. Real-Time Control Technology of 3D Human Model

Controlling the human body model has always been an important direction of virtual reality research. Considering from different aspects to control the virtual human body model, the main methods are as follows: key frame control method, motion capture method, and dynamic method.

The key technology is to study the earliest method of controlling mannequins. The concept of keyframes started with the process of manga animation. In the process of making animation, the superior animator first made the main animation of the comic, which is the so-called key frame, and then the general staff completed the design and realization of the frame in the middle. After that, with the development of computer technology, the generation of the intermediate frame is gradually completed by computer. In animation, the parameters that affect the image of the screen are the parameters that affect the keyframes later.

Due to the particularity of human motion, the best way to use the human body model to express the human motion is to start directly from the motion of the human body. By using the sensor to directly capture the information of each position of the human body, use the parameters obtained by the sensor to reproduce the movement of the human body. Since the parameters obtained in this way are very real human state numbers, it is easy to restore the movement of the human body. However, motion capture technology also has many problems that restrict it to solve all practical applications.

The methods of kinematics are divided into forward kinematics and inverse kinematics. The joints of the virtual human can achieve effective movement through the forward kinematics method and the inverse kinematics method. In cis-kinematics, end-effectors (hands, feet, etc.) are used as a function of time. The position of the end effector is independent of the force or moment causing the action and is resolved by a fixed reference frame. Converting positions and velocities from joint space to Cartesian coordinates is a well-established method. The first application of cis-kinematics was a parametric keyframe animation, where the motion of the joint body was driven by interpolating the major joint angles into the cis-kinematics of the hands and feet. Advanced animators with years of experience can produce very realistic motions by means of cis-kinematics. But it is difficult for ordinary animators to produce realistic motion by setting individual keyframes in combination.

### 3.6. Integrated Manifold Ordering Information Retention

A new manifold supervised dimensionality reduction algorithm is proposed, that is, Integrated Manifold Ordering Information Preservation (EMRP). First, in order to solve the phenomenon of measurement concentration, we need to retain the ranking information of the samples within the class, and in order to extract the discriminative information, we need to maximize the edge distance of the samples between classes. To better understand the difference between method and other manifold supervision methods, this section adopts the PAF framework to construct EMRP.

For a certain recognition problem, *K* samples can be expressed by a matrix composed of fixed-length features:

(1) $$\begin{array}{c} A=\left[a_{1},a_{2},\ldots ,a_{K}\right]\in R^{D\times K}. \end{array}$$

The class of each D-dimensional feature vector *a*_*i*_ ∈ *R*^*D*^ is labeled as

(2) $$\begin{array}{c} Z=\left[z_{1},z_{2},\ldots z_{K}\right]\in C^{K}. \end{array}$$

The purpose of manifold supervised dimensionality reduction learning is to find the projection matrix *U* ∈ *R*^*D*×*d*^ to project the original sample A from the high-dimensional space to the low-dimensional subspace *R*^*d*^, so as to obtain a concise expression:

(3) $$\begin{array}{c} B=U^{S}A=\left[b_{1},,b_{2},\ldots b_{K}\right]\in R^{d\times K}. \end{array}$$

Here, *d* < *D*.

Under the PAF framework, we define an arbitrary sample *a*_*i*_, its intraclass neighbor samples *a*_*i*_1__,…, *a*_*i*_*n*_1___ and *n*_2_ interclass neighbor samples *a*_*i*_1__,…, *a*_*i*_*n*_2___ as a local block:

(4) $$\begin{array}{c} A_{i}=\left[a_{i_{1}},a_{i_{2}},\ldots ,a_{i_{n_{1}}},a_{i_{1}},\ldots ,a_{i_{n_{2}}}\right]\in R^{D\times \left(k_{1}+k_{2}+1\right)}. \end{array}$$

EMRP finds the corresponding low-dimensional expression as

(5) $$\begin{array}{c} B_{i}=\left[b_{i_{1}},b_{i_{2}},\ldots ,b_{i_{n_{1}}},b_{i_{1}},\ldots ,b_{i_{n_{2}}}\right]\in R^{D\times \left(k_{1}+k_{2}+1\right)}. \end{array}$$

The optimization goals on the block include the following:

1. Retain the sorting and retention information between samples within a class;
2. Maximize the discriminative information of between-class samples.

#### 3.6.1. Retention of Sorting Information

The ranking information of the samples within the class is available for classification. Inspired by the LE algorithm, we define the intraclass ordering information on a local block as

(6) $$\begin{array}{c} R\left(b_{i}\right)=\sum_{j=1}^{n_{1}}b_{i}-b_{i^{j}}^{2}{\left(w_{i}\right)}_{j}. \end{array}$$

Here, the weight factor (*w*_*i*_) is defined as

(7) $$\begin{array}{c} {\left(w_{i}\right)}_{j}=\left\{\begin{array}{cc} xp\left(-\frac{a_{i}-a_{i^{j}}^{2}}{s}\right), & e\text{ if }a_{i^{j}}\in K_{n_{1}}\left(a_{i}\right);\;\\ 0 & \text{otherwise} \end{array}\right). \end{array}$$

According to the PAF framework, we can deduce (6) as follows:

(8) $$\begin{array}{c} R\left(b_{i}\right)=\text{tr}\left(B_{R\left(i\right)}L_{R\left(i\right)}B_{R\left(i\right)}^{S}\right). \end{array}$$

Here,

(9) $$\begin{array}{c} L_{R\left(i\right)}=\left[\begin{array}{c} -e_{n_{1}}^{S}\\ I_{n_{1}} \end{array}\right]\text{diag}\left(w_{i}\right)\left[\begin{array}{cc} -e_{n_{1}} & I_{n_{1}} \end{array}\right],\\ e_{n_{1}}={\left[\overset{n_{1}}{\overset{︷}{1,\ldots ,1}}\right]}^{S},\\ I_{n_{1}}=\text{diag}\left[\overset{n_{1}}{\overset{︷}{1,\ldots ,1}}\right],\\ B_{R\left(i\right)}=\left[b_{i},b_{i_{1}},\ldots ,b_{i_{n_{1}}}\right]. \end{array}$$

#### 3.6.2. Maximize Identification Information

For popular supervised learning, discriminative information plays a crucial role. As far as the EMRP algorithm is concerned, we consider that the purpose of extracting discriminative information is achieved by maximizing the distance sum of the samples between *b*_*i*_ and *n*_2_ classes, namely,

(10) $$\begin{array}{c} D\left(b_{i}\right)=\sum_{p=1}^{n_{2}}b_{i}-b_{i_{p}}^{2}{\left(v_{i}\right)}_{j}. \end{array}$$

The definition of the weight factor (*v*_*i*_) here considers the factor of removing the ranking information between classes, namely,

(11) $$\begin{array}{c} {\left(v_{i}\right)}_{j}=\left\{\begin{array}{cc} 1, & \text{if }a_{i^{j}}\in K_{n_{1}}\left(a_{i}\right);\\ 0 & \text{otherwise} \end{array}.\right) \end{array}$$

Under the framework of PAF, we can further derive (10) as

(12) $$\begin{array}{c} D\left(b_{i}\right)=\text{tr}\left(B_{D\left(i\right)}L_{D\left(i\right)}B_{D\left(i\right)}^{S}\right). \end{array}$$

Here,

(13) $$\begin{array}{c} L_{D\left(i\right)}=\left[\begin{array}{c} -e_{n_{2}}^{S}\\ I_{n_{2}} \end{array}\right]\text{diag}\left(v_{i}\right)\left[\begin{array}{cc} -e_{n_{2}} & I_{n_{2}} \end{array}\right],\\ e_{n_{2}}={\left[\overset{n_{2}}{\overset{︷}{1,\ldots ,1}}\right]}^{S},\\ I_{n_{2}}=\text{diag}\left[\overset{n_{2}}{\overset{︷}{1,\ldots ,1}}\right],\\ B_{D\left(i\right)}=\left[b_{i},b_{i_{1}},\ldots ,b_{i_{n_{2}}}\right]. \end{array}$$

Therefore, we can get the optimization objective function on the local block:

(14) $$\begin{array}{c} \arg\min\left(\overset{n_{1}}{\underset{j=1}{\sum }}b_{i}-b_{i^{j}}{}^{2}{\left(w_{i}\right)}_{j}-\gamma \overset{n_{2}}{\underset{p=1}{\sum }}b_{i}-b_{i_{p}}{}^{2}{\left(v_{i}\right)}_{j}\right). \end{array}$$

However, different hyperparameters (such as *n*_1_ in (6) and *n*_2_ in (10)) correspond to manifold with different geometric information, which can seriously affect the final recognition accuracy. In EMPR algorithm, the hyperparameters *s*, *n*_1_, and *n*_2_ that affect the objective function are difficult to choose optimal settings. Therefore, an automatic manifold estimation method is valuable for solving this problem.

### 3.7. Folk Dance

China is a multiethnic country. Every nation has a distinct national culture. Ethnic folk dance originates from life labor and is a dance that people dance to entertain themselves. People express their life through dance and show their unique national charm. The types of Chinese folk dances are shown in Figure 6.

With the changes of the times, ethnic folk dance has gradually evolved into a dance form with its own national characteristics and advancing with the times in the new era on the premise of retaining its original characteristics. It has also gradually expanded from a self-entertainment model to a professional and large-scale system. It is a dance course processed and refined by professional dancers. It is a dance work that expresses ideas in combination with life. The stage sublimation of the national folk dance drama flourished.

Folk dance is the art form of a people who have lived in a specific geographical location for a long time and have developed unique folk customs, religious beliefs, and agricultural civilization. It gradually developed a unique aesthetic taste when combined with the unique natural environment. Ethnic dance can be described as an important cultural carrier that can pass down ancient Chinese folk culture and serves as an external manifestation of national cohesion. Because each ethnic group has its own unique history, rich cultural connotation, and independent national aesthetic habits, each ethnic group has its own dance art language. Folk dance, as a result, has a distinct national character, a limited regional character, and a high level of “self-entertainment.”

Ethnic dance has a long history and is created by workers of all ethnic groups in the context of long-term production practices and life changes. They use innovative dance techniques to convey national history, religious beliefs, life lessons, and even myths and stories. With so many cultural contents, the folk dance is destined to have historical and cultural value, as it is the spiritual wealth left by the forefathers. We can better inherit folk dance by learning it, and we can bring out the functions of cultural inheritance, cultural accumulation, cultural exchange, and cultural innovation of folk dance by learning it.

## 4. Algorithm Data Set Comparison Test Experiment

### 4.1. Dataset Test Experiment

Some images are randomly taken from a subset of the source data and test set LFW, it may be difficult to distinguish where they come from, and the image distributions of the source and target domains are similar.  Table 1 shows experimental results on a subset of the test set LFW dataset.

It can be observed that the model learned in this paper in the source domain is directly tested in the target domain without transfer learning. The results are unsatisfactory, using the cosine and LRA methods to measure the similarity between faces with the lowest results of 82.01% and 85.23%, respectively.

The image distributions of the source and target domains are quite different. Considering the variation of expression, illumination, and occlusion, restricted parameter learning method RPL shows its superiority in the FERET dataset.

Two 2048-dimensional representative feature vectors are concatenated to a 4096-dimensional feature vector without principal component analysis (PCA) dimensionality reduction for face recognition. The similarity between features is then measured with the LRA method. The results of the RPL method in this paper on the two databases and the comparison results of other methods and other recent works are shown in Table 2.

All in all, using the restricted parameter learning (RPL) deep transfer learning method, the learning space of parameters in the target domain is constrained. By adjusting the source domain knowledge of the scarce target domain samples, overfitting and parameter structure damage can be prevented, and ideal results can be obtained in the same and different distributions. Unlike other state-of-the-art techniques, method can adjust knowledge from the source domain to the target domain offline; that is, it does not require training on both source and target data simultaneously. Therefore, the RPL method in this paper can be easily applied to many scenarios. The results validate the effectiveness of RPL, which uses very deep convolutional networks fine-tuned with sample knowledge in the target domain.

### 4.2. Algorithm Dataset Comparison Experiment

Figure 7 shows the best average recognition rate of the test set for the six algorithms under different training samples on the NMHA-TP dataset (including two cases of *p* = 20 and *p* = 30).

It can be seen that, compared with several other algorithms, the EMPR algorithm can obtain the best classification performance on the NMHA-TP dataset.

Figure 8 shows the best average recognition rate of the six algorithms in the test set under different training samples on the NMHA-WP dataset (including two cases of *p* = 20 and *p* = 30).

It can be seen that, compared with several other algorithms, the EMPR algorithm can obtain the best classification performance on the NMHA-WP dataset.

Table 3 presents the best average recognition rates and corresponding dimensions of the six algorithms on the NMHA-TP-WP dataset.

It can be seen that, compared with several other algorithms, the EMPR algorithm can obtain the best classification performance on the NMHA-TP-WP dataset.

In addition, Table 4 shows the comparison results of the six algorithms and the RPDA algorithm on the SCUTNAA dataset. It can be seen that the EMRP algorithm has a certain advantage in the recognition rate compared with the RPDA algorithm. In addition, the experimental results of EMRP-81 and EMRP-9 show that more candidate matrices are helpful for the learning of the essential manifold.

The main conclusions of the EMRP-related experiments can be summarized as follows:

1. Algorithms such as EMRP, RPDA, LSDA, and MFA are suitable for human action recognition based on acceleration sensor due to the intuitive consideration of the geometric information on the local block. The EMRP and RPDA algorithms perform better because of considering the balance between the ranking information of the intraclass neighbor samples and the neighbor ranking information of the interclass samples.
2. In the human action recognition test based on the acceleration sensor of mobile phone, EMRP-81 significantly improves the recognition accuracy and obtains the best average recognition rate. All of these demonstrate the robustness and effectiveness of the EMRP algorithm in the human action classification task. This also proves that the EMRP-based algorithm can learn a linear combination of candidate registration matrices to obtain better system performance.

### 4.3. Comparison Experiment of Target Matching Algorithms

The VOT dataset and six representative image sequences from the TempleColor128 dataset are used to evaluate the algorithm in this paper. The Juice image sequence is specifically included. The target has a slight spatial transformation, while the background has a small spatial transformation. The background in this data changes dramatically, the target is scaled and rotated, and there is also similar target interference. There are severe illumination changes in this data, as well as deformation in the target itself, in the motorcycle image sequence. The target in this data has scale, illumination, and certain morphological transformations, as seen in a helicopter image sequence. The shape of the target changes, the background changes slightly, and there is partial occlusion in this data from a skier image sequence. In this data, there are similar targets, the target has large deformation and scale transformation, and the background also has transformation. After manually culling the images whose targets were completely occluded and difficult to identify in the image sequence, about 10 images were selected as training data, and other images were used as test data in the experiment. The intersection ratio, recall, and efficiency of the four algorithms on six groups of image sequences are shown in Figure 9.

According to the experimental data, it can be seen that the traditional algorithm only has good results in some scenarios, while the method based on machine learning can take into account most scenarios.

The grayscale template matching based on the correlation coefficient has a good effect on simple scenes such as Juice image sequences and also has a good effect on scenes with simple backgrounds and small target deformation, such as Skier and Crossing image sequences. However, the target matching performance of these scenes depends on the influence of template selection, which is not very stable. Only when the template is selected properly, there is a better matching effect. The overall performance is not very stable.

The algorithm based on SIFT registration has better performance in simple scenes such as Juice image sequences, but when the target is deformed, or the imaging quality is poor, the matching effect is obviously degraded. The overall performance is poor.

The algorithm based on feature template also performs well in simple scenes, but when the scene is complex, the performance deteriorates, and the algorithm's intersection and union are relatively low, and the matching accuracy is poor. And the overall performance is poor.

## 5. Comparative Analysis of Few-Shot Learning for 3D Digital Modeling of Folk Dance Based on Gesture Recognition

The algorithm data set is analyzed through experiments, and finally the Few-Shot learning method for 3D digital modeling of folk dance based on gesture recognition designed in this paper is optimized. In order to verify how this Few-Shot method is different from traditional learning methods for folk dance learning, this paper designs a set of comparative experiments. In this paper, 20 students majoring in folk dance are divided into two groups. One group uses the Few-Shot learning method designed in this paper based on the three-dimensional digital modeling of folk dance based on gesture recognition. The other group used traditional folk dance learning methods and then judged their learning efficiency based on the learning time and movement scores of the two groups of students. The experimental data is shown in Figure 10.

As can be seen from Figure 10, the time for students majoring in ethnic dance to learn the Few-Shot learning method based on gesture recognition 3D digital modeling of ethnic dance designed in this paper is only 8.93 minutes for the same dance. The time used in the traditional folk dance learning method is 10.77 minutes. Compared with the traditional learning method, the Few-Shot learning method based on gesture recognition 3D digital modeling of folk dance designed in this paper reduces the learning time by 17%. And the dance action score of the Few-Shot learning method designed in this paper reaches 92.96 points, while the traditional learning method is only 81.46 points. It can be seen that the Few-Shot learning method designed in this paper is 14% higher than the traditional learning method. To sum up, the Few-Shot learning method based on gesture recognition and three-dimensional digital modeling of ethnic dance designed in this paper can effectively improve the learning efficiency of ethnic dance students majoring in ethnic dance.

## 6. Conclusion

This paper mainly studies the 3D digital model of folk dance based on Few-Shot learning and gesture recognition. Therefore, this paper combines the human body detection and tracking technology of human body posture recognition technology to collect the movement posture and human body posture data of folk dance. Then, this paper uses the AAM model to perform 3D digital modeling of the collected action poses. Then, this paper retains by integrating the manifold ordering information and finally designs a folk dance learning method combined with the Few-Shot learning method. This paper also designs a data set test experiment and an algorithm data set comparison experiment to optimize the algorithm test and data set design. Then, this paper carries out the final optimization according to the experimental results of the target matching algorithm comparison experiment. This paper designs a Few-Shot learning method for 3D digital modeling of folk dance based on gesture recognition. This method can scientifically and effectively improve the learning efficiency and performance of students majoring in ethnic dance.

## Figures and Tables

**Figure 1:** Principle of structured light collection.

**Figure 2:** The principle of time-of-flight acquisition.

**Figure 3:** Motion capture system.

**Figure 4:** Piecewise affine transformation.

**Figure 5:** Calculation process of piecewise linear affine transformation.

**Figure 6:** Types of Chinese folk dances.

**Figure 7:** Best Average Recognition Rate of 6 Algorithms on NMHA-TP Dataset (a) *p* = 20 (b) *p* = 30.

**Figure 8:** The best average recognition rate of the six algorithms on the NMHA-WP dataset (a) *p* = 20 (b) *p* = 30.

**Figure 9:** Comparison of experimental results of target matching algorithms. (a) Cross-comparison experimental results. (b) Recall experiment results. (c) Effectiveness experimental results.

**Figure 10:** Comparison of learning efficiency between the few-shot learning method designed in this paper and the traditional learning method. (a) Study time comparison. (b) Action score comparison.

**Table 1:** Test results on LFW dataset.

methods	ACC (%)	Methods	ACC (%)
Ws + cos	82.01	Ws + LRA	85.23
Pure + cos	84.52	Pure + L RA	87.87
RPL (L1) + cos	85.98	RPL (L1) + L/RA	88.91
RPL (L2) + cos	88.70	RPL (L2) + LRA	89.33

**Table 2:** Results of multiregion feature fusion.

Feret	fb	fc	dup1	dup2	Ave
G-LQP	99.9	100	93.2	91	96.03
LGBP-LGXP	99	99	94	93	96.25
sPOM + POD	99.7	100	94.9	94	97.15
GOM	99.9	100	95.7	93.1	97.18
PCANet2	99.58	100	95.43	94.02	97.26

**Table 3:** The best average recognition rate of the six algorithms on the NMHA-TP-WP dataset.

algorithm	PCA	LDA	L SDA	MFA	GMSS	EMRP-9	EMRP-81
Falling	0.770	0.706	0.771	0.671	0.692	0.739	0.785
Jumping	0.849	0.860	0.850	0.795	0.821	0.910	0.911
Running	0.901	0.876	0.868	0.898	0.898	0.953	0.955
Sit to stand	0.588	0.584	0.558	0.611	0.485	0.606	0.585
Stand to sit	0.619	0.608	0.658	0.671	0.440	0.702	0.695
Walking	0.682	0.663	0.706	0.763	0.768	0.768	0.792
Step walking	0.859	0.882	0.965	0.932	0.950	0.924	0.937

**Table 4:** Comparison of RPDA algorithm and 6 algorithms on SCUT NAA dataset.

number Of training samples	*P* = 20							
Algorithm	PCA	LDA	LSDA	MFA	GMSS	RPDA	EMRP-9	EMRP-81
Average accuracy	0.732	0.736	0.751	0.755	0.767	0.773	0.778	0.780
Dimensionality reduction	(30)	(8)	(7)	(9)	(5)	(27)	(27)	(28)

## Data Availability

The data used to support the findings of this study are available from the corresponding author upon request.
